# Application of Wireless Network Multisensor Fusion Technology in Sports Training

This article has been retracted.

**DOI:** 10.1155/2022/9836697

**Published:** 2022-06-03

**Authors:** Wenjun Tang

**Affiliations:** PE Department of Tongling University, Tongling 244061, Anhui 244061, China

## Abstract

Fencing is an advantageous event for a country to participate in the Asian Games. The discussion and research on the means and methods of special fencing ability training are of great significance to the further development of fencing in the country. Based on the multisensor information fusion technology, this paper develops a special fencing training system with digital monitoring and intelligent decision-making. The multisensor information fusion technology scheme, which is reported in this paper, is used to perform decision-level fusion based on fuzzy inference technology whereas Kalman filter is used to optimize the original information. On the basis of the overall structure, mechanical mechanism, and performance analysis, the mechanical prototype of the fencing special ability training system was developed whereas design, processing, and debugging of the prototype were completed. Combined with the mechanical prototype design of various index parameter display structures based on multisensor information fusion technology, the digital processing of the fencing special ability training system is realized. The force, speed, position, and other characteristic quantities in the fencing special training system are collected by the pressure and rotational speed sensors respectively whereas USB communication technology is used for data transmission. On the basis of in-depth analysis of the characteristics of the special training system for fencing, an abstract system of pedaling power based on the center of gravity and trend models is designed where the Kalman filter is reserved for the special application fields. Moreover, the core role of Kalman filter is carried out when original data information is needed to be obtained. By constructing a force distribution pressure center trajectory measurement model, a training load and training parameter measurement model, and a training level evaluation model, the data-level raw information is specially processed to generate more training parameters that meet specific characteristics, making the multisensor information fusion technology more efficient. It is well integrated into the fencing special ability training system. By applying fuzzy reasoning technology, the special training parameters and the relationship between these parameters are transformed into fuzzy sets and fuzzy rules, and the perceptual knowledge of sports training experience is transformed into fuzzy rules. With this decision-level data fusion method, the fencing special training system has certain intelligent functions.

## 1. Introduction

In the process of multisensor fusion, due to the uncertainty of the fusion information, it cannot be directly classified or adopt clear rules. Therefore, this paper adopts the fuzzy logic inference method and uses the domain of discourse, membership function, and other means to establish the fusion information. Uncertainty is described, and then the corresponding fusion results are obtained in the fuzzy logic reasoning process. In fact, a complex nonlinear mapping relationship between the multisensor output data space and the target data space is realized in the inference process, and such a nonlinear mapping relationship has strong fault tolerance and robustness. Unlike the Kalman filter method, this method does not require an accurate mathematical model, avoiding the bias caused by the inaccurate model of the system.

When selecting a training load for a certain training method, it is difficult for the coach to adjust the training load in a timely and accurate manner according to the current situation of the athlete. To solve this problem, it is necessary to develop an intelligent system with training load navigation ability. Decision-level data fusion effectively combine various information source such as data, interpret the meaning of training parameters according to training experience, and make target diagnostic information more accurate. This is the research motivation for applying fuzzy inference fusion technology. The goal of decision-level data fusion research is to improve the decision-making performance of the system by imitating the diagnostic ability of sports training experts.

Fuzzy knowledge about sports training is the characterization of perceptual knowledge based on training experience. Based on the characteristics of coaches and athletes identifying and judging complex training phenomena, fuzzy mathematical concepts are established. Based on fuzzy linguistic variables or fuzzy algorithms, fuzzy theory provides an approximate, effective, and more flexible method for describing system behavior for complex systems that are difficult to analyze mathematically. This paper adopts the idea of fuzzy reasoning, which is to transform the knowledge and experience of training experts into the form of language rules in the form of IF-THEN, avoiding complex mathematical operation models. In the special ability training system, the training load plays an important role in the special ability training, and the change of the athlete's training load has a great influence on the development of the special ability. The decision-level information fusion technology is applied to the training load diagnosis system. By monitoring various training parameters in real time, after the fusion processing of the fusion center, the complementarity of multisource information is fully utilized, thereby enhancing the reliability of training load diagnosis. The evaluation performance of the training target decision system is improved.

Initially, this paper tries to conduct evaluation of the special training level and then training target decision-making functions, which are primarily based on multisensor information fusion technology. In the information fusion method, fuzzy reasoning technology is one of the effective solutions to the problem and generates more valuable information through its fusion ability. In addition, the decision-level data fusion process does not exist independently but is an organic part of the special ability training system based on multilevel data fusion technology.

The rest of the manuscript is arranged according to the description that is provided in the paragraph given below.

In the subsequent section, training activity of the required or expected target decision-making function is defined and explained with supportive literature review contents. Training load target monitoring method is described in Section 3 of the paper.  Section 4 is dedicated to training load target decision process whereas the subsequent section has described experimental analysis of training load target decision-making which is followed by the concluding remarks.

## 2. Analysis of Training Target Decision-Making Function

In order to preliminarily realize the function of special training level assessment and training target decision-making based on multisensor information fusion technology, it is first necessary to clarify the monitoring tasks of the special fencing training system. The special ability of fencers is the main factor affecting the performance of the competition [1]. Therefore, the special training load and its optimization have become more and more concerned in the fencing industry, and the establishment of a load monitoring and optimization model is of great significance to improve the special ability. The key issue is how to transform the initially processed sensor data into information and knowledge to support decision-making in a timely manner [2, 3]. This involves how to reasonably utilize various feature information to construct an evaluation model. By extracting the characteristic training parameters from the information obtained by each sensor and analyzing the special meaning and purpose, the decision support data of the system is identified and input to the fuzzy inference system for decision-level fusion.

Due to the ambiguity and variability of wind resistance loads generated by different pedaling forces of different athletes, it is difficult to define and correlate them. The traditional method of grading wind resistance load is difficult to reflect the changes of various factors. It is reasonable to determine the load intensity. It is not easy to determine the boundary [4]. Assuming that 20 units are the boundary, then 21 units are defined as “reasonable,” and 19 units are defined as “poor,” which is unscientific. Importantly, there is also ambiguity in the quality of training produced by windage loads. The function to be realized by the training target decision system is to adjust the current load in real time by comparing the target amount of the training load with the current amount. In the training load detection and prompting mode, the fusion center can identify the training load trajectory trend and nature. The first function is to establish a fuzzy relationship matrix so that the training target decision-making system has the ability to navigate training parameters so as to realize the increase or decrease of the training load around the optimal load trajectory through the athlete. Referring to Figure 1, if the load trajectory fluctuates greatly, reduce the load by reducing the speed and resistance (the technical action remains unchanged, and the standardization of the special ability is guaranteed). If the load trajectory fluctuation is small, increase the load amount.

See Table 1; this is the fuzzy inference rule for special ability training aiming at maintaining a certain degree of load trajectory fluctuation.

Usually, an athlete's training program is cyclical in nature, with the goal of gradually adapting the body to the ability and level of the competitive state. Therefore, establishing the optimal relationship between training objectives, training content, training phases, and training load requires a balance between appropriateness and complementarity. This requires intelligent decision-making results to provide multiple types of decision-making services [5] and adopt different decision-making services for different monitoring results. The information provided by the qualitative factors of the athlete's training ability needs to be taken into account so that more positive results can be obtained. According to the scientific index system, the ability to complete the training load and the degree of trustworthiness of the rated athletes are objectively and impartially evaluated by concise text symbols, and the load intensity is analyzed by the fuzzy reasoning method, and the load capacity level is determined [6].

The purpose of decision-level fusion is to build an evaluation model, not a control model—control itself is the athlete's initiative. The goal of the intelligent system is to keep the load trajectory stable within the desired range. Using fuzzy technology to design a decision-making assistance system, it can process digital information and describe the system behavior with language rules, simulate the trainer's reasoning and decision-making process through fuzzy logic, predict the change of load trajectory, and assist the trainer to make decisions about the change of training load [7].

Referring to Figure 2, it is assumed that the load trajectory changes according to a certain trend and pattern. With the change of training requirements, the training parameter indication is generated by the inference engine, and the athlete activates another more suitable movement trend and pattern according to the indication information. Efficiently meet training requirements.

Through the tracking and diagnosis of the load trajectory under a certain training level, the optimal training parameter results are determined by the fuzzy reasoning engine. Control the training load to track the training target within a certain optimized range.

## 3. Training Load Target Monitoring Method

According to the above fuzzy reasoning method, the current load capacity level of the athlete can be diagnosed. Conversely, training requirements are adjusted according to the training plan. Additionally, when the training load needs to be kept at the *n*th level [8, 9], the specified ranges of the training parameters related to the positional and velocity properties are obtained according to the rule base and the membership function.

Referring to Table 2, the training parameter set corresponding to the training load level is: *S* = {*s*_1_, *s*_2_, *s*_3_} = {push amplitude, pedal frequency, pedal force}. For example, the athlete is required to carry out the third-level load training, and the position and speed are at a moderate level [10]. According to the definition of the corresponding member function, the training parameter related to the position is that the pedaling amplitude is kept between 1 and 1.5, and the speed is different. The relevant training parameter is to keep the pedaling frequency between 2 and 3.

Referring to Figure 3, when the training load trajectory deviates from the optimal range, start each training parameter monitoring program to monitor the fluctuations of each training parameter—pedaling amplitude, pedaling force, and pedaling frequency—and calculate them according to the fuzzy control rules. The results indicate the amount of modulation for each training parameter. The training load taken by the athlete must maintain a certain load capacity level, and a corresponding training level is required. Adjust and optimize the training parameters according to the difference between the training target intensity of the athlete under a certain training level and the evaluation intensity of the actual load trajectory tracking and diagnosis. Based on the positional training load, the athlete must first ensure the specialization of the training load through the pedaling range [11] and then adjust the pedaling force and frequency to keep the training load within the optimal range of a certain level. In this way, it is necessary to monitor the level of training load and then monitor the volatility of the training load under a certain level of guarantee. The fuzzy inference method is adopted to adjust the training parameters according to certain training load requirements.

## 4. Training Load Target Decision Process

The real-time assessment of training load capacity is very important to achieve more ideal training quality control. The task of training load target decision-making is coach's assistance to more effectively judge and arrange the training load status of athletes. Through fuzzy decision-making (defuzzification), clear training parameter instructions are obtained [12], and athletes make corresponding adjustments through feedback information to control the training load level within a certain range, thereby scientifically improving training efficiency.

According to the training level evaluation model, the smaller the fluctuation of training parameters under a certain load level, the higher the training level of the athlete. Based on the experience of the coaches, the control rules can be described in words as follows:

The greater the volatility, the greater the change in adjusting the training parameters; otherwise the change is small. The difference *e* between the training load or the current amount of training parameters and the target amount reflects the volatility, and the fuzzy set of language values is {negative large, negative small, zero, positive small, positive large}, denoted as NB = negative large, NS = negative small, *O* = zero, PS = positive small, and PB = positive large.

Let the universe of discourse of load deviation *e* be *X* and quantify it into 7 levels:

(1) $$\begin{array}{c} X=\left\{-3,-2,-1,0,1,2,3\right\}. \end{array}$$

The domain of a certain training parameter regulation *u* is *Y*, and like *X*, it is also divided into 7 levels; see Table 3:

(2) $$\begin{array}{c} Y=\left\{-3,-2,-1,0,1,2,3\right\}. \end{array}$$

See Figure 4 for membership function curves with linguistic variables.

A fuzzy control rule is actually a set of multiple conditional statements, which can be expressed as a fuzzy relation *R* from the bias universe *X* to the regulating quantity universe *Y*. When the domain of discourse is limited, the fuzzy relationship can be represented by a matrix [13]. See Table 4.

The negative large deviation is expressed as *NB*_*e*_, and the corresponding positive large control amount is expressed as *PB*_*u*_. The difference between the deviation and the control amount is.

In a similar situation, there is

(3) $$\begin{array}{c} R=\left(NB_{e}\times PB_{u}\right)+\left(NS_{e}\times PS_{u}\right)+\left(O_{e}\times O_{u}\right)+\left(PS_{e}\times NS_{u}\right)+\left(PB_{e}\times NB_{u}\right),\\ R=\left[\begin{array}{ccccccc} 1 & 1 & 1 & 1 & 0 & 0.6 & 1\\ 0 & 0 & 0 & 0 & 1 & 1 & 0.4\\ 0 & 0 & 0.2 & 0.5 & 0.5 & 1 & 1\\ 1 & 0 & 0.4 & 1 & 0.4 & 0.4 & 0\\ 0 & 0.1 & 1 & 0.6 & 0.9 & 0.2 & 0.6\\ 0.4 & 0.3 & 0.2 & 1 & 0 & 0.1 & 0.3\\ 1 & 0.7 & 0.3 & 1 & 0 & 0 & 1 \end{array}\right]. \end{array}$$

The control quantity *u* is actually equal to the synthesis of the fuzzy vector of the deviation and the fuzzy relation *R*. When the bias is *PS*, there is *u*=(0.5, 0.5, 1,0.5, 0.5, 0,0). For the fuzzy subset of the control variable, according to the principle of maximum membership, the control variable should be selected as “−1” level; that is, when the deviation is PS, the control variable is qualitatively NS.

There are three fuzzy subsets: [low], [medium], and [high] on the pedaling frequency, pedaling amplitude, and pedaling force energy universe. The membership of the actual value to the fuzzy subset is determined according to the membership function. For example, when the actual value *w*_0_=1, *f*_0_=2.5, *F*_0_=1.25, *q* = 0.9 time, [ low ](*w*_0_) = 0.5 ，[ middle ](*w*_0_) = 0.5, [ high ](*w*_0_) = 0; [ low ](*f*_0_) = 0, [ middle ](*f*_0_) = 1, [ high ](*f*_0_) = 0, [ Low ](*F*_0_) = 0¸[ middle ](*F*_0_) = 1¸[ high ](*F*_0_) = 0. Referring to Table 5, the training load level is evaluated by the fuzzy rules of types A and B.


(4) Z=A∑i=19μAiz×leveli∑i=19μAiz=0.5×2+0.5×3=2.5,ZB=∑i=19μBiz×leveli∑i=19μBiz=0.5×2+1×3=3.5,Z0=qa×ZA+qb×q×ZBqa+qb×q=0.5×2.5+0.5×0.9×3.50.5+0.5×0.9=2.97.

Therefore, the actual training load level based on the A-type fuzzy rules is level = 2.5. The comprehensive fusion result considering the influence of B-type fuzzy rules is level = 2.97.

See Figure 5, which lists the relationship between the pedaling amplitude and the pedaling frequency under the load levels 1.5, 2, 2.5, 3, 3.5, 4, and 4.5.

Under a certain training load level, the regulation sequence of each training parameter is pedaling amplitude ⟶ pedaling frequency ⟶ pedaling power because first of all, it is necessary to sacrifice the stability of the pedaling force to gradually obtain the stability of the pedaling amplitude and the pedaling frequency, and finally adjust the pedaling force [14–16]. If the training requires changing the load level, you can increase the pedaling range while maintaining the current pedaling frequency and then increase the pedaling frequency while maintaining the new pedaling range to gradually reach the required training load level.

If the training requirement controls the training load level to level = 3.5, according to the fuzzy rules based on class A.

The fuzzy relationship between the load level, the pedaling amplitude and the pedaling frequency, and a certain pedaling amplitude corresponds to a certain pedaling frequency. Corresponding to a certain training load level, there are various combinations of pedaling amplitude and pedaling frequency, and each pair of pedaling amplitude and pedaling frequency corresponds to a certain pedaling force [17]. Under the condition of different pairs of pedaling frequency and pedaling amplitude, the pedaling force of the athlete is different. The power of pedaling is the cause of the reaction of wind resistance and rotational speed, which is expressed in the form of force or work in physical energy consumption. According to the principle of the minimum pedaling force and the maximum pedaling quality coefficient, the combination of pedaling frequency and pedaling amplitude is optimized, and the fusion result based on the fuzzy rules of class A and class B approaches the target level = 3.5. In this way, the optimization of load trajectory includes two conditions: the principle of force minimization and the principle of specialization so that the pertinence and scientificity of athletes' special ability training can be further developed [18].

## 5. Experimental Analysis of Training Load Target Decision-Making

Assuming that the training task of level 0 = 3.5 load is carried out, the pedaling amplitude according to the requirements of the training program is *w*_0_=1.3, and the pedaling frequency is *f*_0_=2.9. The athlete regulates and stabilizes the pedaling amplitude and the pedaling frequency according to the instructions of the training parameters.

Make the load level deviation *e*_level_=level − level_0_, pedaling power deviation *eF*=*F* − *F*_min_, where *F*_min_ is the smallest one-time average pedal effort in the continuously updated training task history. Athletes refer to *F*_min_ for optimal regulation of pedaling power.

This defines the relative value of the deviation and the target amount *e*%=*e*_level_/level_0_. Above 10% is 3rd gear, (5%, 10%] is 2nd gear, (2%, 5%] is 1st gear, [−2%, 2%] corresponds to 0th gear, [−5%, −2%) corresponds to −1 gear, [−10%, −5%) corresponds to −2 gear, and below −10% corresponds to −3 gear.

As shown in Figure 6, during the actual operation of the system, the load level deviation *e*_level_ is detected, and the deviation fuzzy vector is formed, which is synthesized with the fuzzy relationship matrix *R* to obtain the corresponding control amount, as shown in Figure 7.

When −10 ≤ *e*%≤−3, the membership degree of the corresponding element in the universe is

(5) $$\begin{array}{c} \mu_{\left(-1\right)}\left(e\%\right)=\frac{10\%+e\%}{10\%-3\%},\\ \mu_{\left(-2\right)}\left(e\%\right)=\frac{4.5\%-\left|e\%+7.5\%\right|}{7.5\%-3\%},\\ \mu_{\left(-3\right)}\left(e\%\right)=\frac{-3\%+e\%}{10\%-3\%}. \end{array}$$

When −7.5 ≤ *e*%≤0, the membership degree of the corresponding element in the universe is

(6) $$\begin{array}{c} \mu_{\left(0\right)}\left(e\%\right)=\frac{7.5\%+e\%}{7.5\%}. \end{array}$$

When −3 ≤ *e*%≤0, the membership degree of the corresponding element in the universe is

(7) $$\begin{array}{c} \mu_{\left(-1\right)}\left(e\%\right)=\frac{-e\%}{3\%}. \end{array}$$

When 0 ≤ *e*%≤3%, the membership degree of the corresponding element in the universe is

(8) $$\begin{array}{c} \mu_{\left(1\right)}\left(e\%\right)=\frac{e\%}{3\%}. \end{array}$$

When 0 ≤ *e*%≤7.5%, the membership degree of the corresponding element in the universe is *μ*_(0)_(*e*%)=7.5%−*e*%/7.5%.

When 3 ≤ *e*%≤10%, the membership degree of the corresponding element in the universe is

(9) $$\begin{array}{c} \mu_{\left(1\right)}\left(e\%\right)=\frac{10\%-e\%}{10\%-3\%},\\ \mu_{\left(2\right)}\left(e\%\right)=\frac{4.5\%-\left|e\%-7.5\%\right|}{7.5\%-3\%},\\ \mu_{\left(3\right)}\left(e\%\right)=\frac{e\%-3\%}{10\%-3\%}. \end{array}$$

For a certain *e*%=3.5%, there are

(10) $$\begin{array}{c} \left(\left({}_{\left(-3\right)}\left(e\%\right)\right)\mu_{\left(-2\right)}\left(e\%\right)\left(\mu_{\left(-1\right)}\left(e\%\right)\right)\mu_{\left(0\right)}\left(e\%\right)\left(\mu_{\left(1\right)}\left(e\%\right)\right)\left(\mu_{\left(2\right)}\left(e\%\right)\right)\mu_{\left(3\right)}\left(e\%\right)\right)\\ =\left(0,0,0,0.53,0.93,0.11,0.07\right). \end{array}$$

The synthetic result with the fuzzy matrix *R* is (0.11, 0.5, 0.93, 0.53, 0.5, 0, 0), and the element with the largest membership degree in the fuzzy set is selected as the final result control amount, which is NS [19].

The training parameter indication fed back to the athlete is opposite to the deviation, and then the fuzzy regulation amount is converted into the adjustment amount of the pedaling amplitude and the pedaling frequency, thereby instructing the athlete to adjust the training parameters as shown in Figure 8.

The current load level is level=(1+3.5%)level_0_=3.6635, and the relevant training parameters need to be adjusted to reduce it to the target load level level_0_=3.5.

Set the current value of the pedaling frequency *f*_*t*_ unchanged, and calculate the fuzzy adjustment amount of the pedaling amplitude as Δ*w*_*t*_=−3.5%*w*_*t*_. The two training parameters are processed synchronously and continuously updated to give the indicated value. In this process, the athlete continuously adjusts the training parameters in the order of pedaling amplitude ⟶ pedaling frequency ⟶ pedaling force, gradually stabilizes to the load target, and optimizes the pedaling force to minimize the pedaling force and the highest possible pedaling force. The pedaling quality coefficient is used to complete the training task, thereby improving the special training ability.

The following is an example of the main points of some software program source code for load level monitoring.

  'Regarding the database definition, save the collected or read data
  'Related training parameters and load level variables, dynamic array definitions
  'About the data variable initialization function
  “Private Sub load level()”load level monitoring function
  For *i* = 1 To 3′ variable array initialization
  Vload_*f*(*i*) = 0; load_*w*(*i*) = 0; load_s(*i*) = 0
  Next
  'Push frequency membership
  If load_*f*(0) ≤  2.5 Then 'low membership
  load_*f*(1) = 2.5 -load_f(0) If load_*f*(0) ≤  1.5 Then load_*f*(1) = 1 End If
  End If
  If load_*f*(0) ≥  2.5 And load_*f*(0) ≤  3.5 Then “ membership in ”
  load_*f*(2) = 3.5 - load_f(0) End If
  If load_*f*(0) ≥  1.5 And load_*f*(0) ≤  2.5 Then
  load_*f*(2) = load_*f*(0) - 1.5 End If
  If load_*f*(0) ≥  2.5 And load_*f*(0) ≤  3.5 Then 'High degree of membership
  load_*f*(3) = load_*f*(0) -2.5 End If
  If load_*f*(0) ≥  3.5 Then load_*f*(3) = 1 End If
  'Push amplitude membership
  If load_*w*(0) ≤  1.25 Then 'low membership
  load_*w*(1) = 2.5–2 *∗* load_*w*(0)
  If load_*w*(0) ≤  0.75 Then load_*w*(1) = 1 End If
  End If
  If load_*w*(0) ≥  1.25 And load_*w*(0) ≤  1.75 Then “ membership in ”
  load_*w*(2) = 3.5–2 *∗* load_*w*(0) End If
  If load_*w*(0) ≥  0.75 And load_*w*(0) ≤  1.25 Then
  load_*w*(2) = 2 *∗* load_*w*(0) -1.5 End If
  If load_*w*(0) ≥  1.25 And load_*w*(0) ≤  1.75 Then 'High degree of membership
  load_*w*(3) = 2 *∗* load_*w*(0) -2.5 End If
  If load_*w*(0) ≥  1.75 Then load_*w*(3) = 1
  End If
  'Pegging power membership
  If load_s(0) ≤  1.25 Then 'low membership
  load_s(1) = 2.5–2 *∗* load_s(0) If load_s(0) ≤  0.75 Then
  load_s(1) = 1 End If End If
  If load_s(0) ≥  1.25 And load_s(0) ≤  1.75 Then ' membership in
  load_s(2) = 3.5–2 *∗* load_s(0) End If
  If load_s(0) ≥  0.75 And load_s(0) ≤  1.25 Then
  load_s(2) = 2 *∗* load_s(0) -1.5 End If
  If load_s(0) ≥  1.25 And load_s(0) ≤  1.75 Then 'high degree of membership
  load_s(3) = 2 *∗* load_s(0) -2.5 End If
  If load_s(0) ≥  1.75 Then load_s(3) = 1
  End If
  loadA(1) = load_*w*(1) *∗* load_*f*(1) 'low-low combination
  load1 = load_*w*(1) *∗* load_*f*(2) 'low and medium combination
  load2 = load_*w*(2) *∗* load_*f*(1) 'Medium and low combination
  If load1 > load2 Then 'take the maximum degree of membership
  loadA(2) = load1 Else loadA(2) = load2 End If
  load1 = load_*w*(1) *∗* load_*f*(3) 'Low and high combination
  load2 = load_*w*(2) *∗* load_*f*(2) 'Combination in the middle
  load3 = load_*w*(3) *∗* load_*f*(1) 'The combination of high and low
  If load1 > load2 Then If load1 > load3 Then
  loadA(3) = load1 Else loadA(3) = load3 End If
  Else If load2 > load3 Then loadA(3) = load2
  Else loadA(3) = load3 End If End If
  load1 = load_*w*(2) *∗* load_*f*(3) 'Medium and high combination
  load2 = load_*w*(3) *∗* load_*f*(2) 'High school combination
  If load1 > load2 Then 'take the maximum degree of membership
  loadA(4) = load1 Else loadA(4) = load2 End If
  loadA(5) = load_*w*(3) *∗* load_*f*(3) 'High and high combination
  load1 = 0; load2 = 0
  For *i* = 1 To 5
  load1 = load1 + loadA(*i*) *∗i*; load2 = load2 + loadA(*i*)
  Next
  loadA(0) = load1/load2
  loadB(1) = load_s(1) *∗* load_f(1) 'low-low combination
  load1 = load_s(1) *∗* load_f(2) 'low and medium combination
  load2 = load_s(2) *∗* load_f(1) 'Mid and low combination
  If load1 > load2 Then 'take the maximum degree of membership
  loadB(2) = load1 Else loadB(2) = load2 End If
  load1 = load_s(1) *∗* load_f(3) 'The combination of low and high
  load2 = load_s(2) *∗* load_f(2) 'Combination in the middle
  load3 = load_s(3) *∗* load_f(1) 'The combination of high and low
  If load1 > load2 Then If load1 > load3 Then loadB(3) = load1
  Else loadB(3) = load3 End If Else If load2 > load3 Then loadB(3) = load2
  Else loadB(3) = load3 End If End If
  load1 = load_s(2) *∗* load_*f*(3) 'Medium and high combination
  load2 = load_s(3) *∗* load_*f*(2) 'High school combination
  If load1 > load2 Then 'take the maximum degree of membership
  loadB(4) = load1 Else loadB(4) = load2 End If
  loadB(5) = load_s(3) *∗* load_f(3) 'High and high combination
  load1 = 0; load2 = 0
  For *i* = 1 To 5
  load1 = load1 + loadB(*i*) *∗i*; load2 = load2 + loadB(*i*)
  Next
  loadB(0) = load1/load2
  load = (loadA(0) + loadB(0) *∗* s_good)/(1 +  *s*_good) '…
  End sub

As shown in Figure 9, according to the training cycle arrangement and special ability needs, the coach proposed that the training load level should be controlled as level = 2.2, the pedaling frequency for strength endurance training is *f* = 1.8, and the corresponding pedaling amplitude is *w*=1.2.

During the actual operation of the system, various training parameters fluctuate randomly within a certain range; for example, the quality coefficient of pedaling power fluctuates around 0.9. The fluctuations of these training parameter indicators interact with each other, which is a fuzzy relationship with the training load level as the goal. The athlete adjusts the changes of relevant training parameters in a timely manner according to the feedback navigation instruction information to stabilize it within the area corresponding to the target load level [20]. When the fluctuations of various training parameters under a certain training load level gradually decrease and become stable, it means that the training level of the athlete's current load level has improved. According to the training target decision, the fuzzy control amount of various training parameters is judged under a certain training load target level, and after various training parameters are adjusted to meet the training load target level, the training level corresponding to the volatility of various training parameters can also be adjusted. Assess the situation, prompting coaches and athletes to increase the training load level intensity and enter a more advanced dynamic balance training mechanism. This cycle, with this digital and intelligent training mechanism, enables athletes to continuously improve their special ability levels in efficient scientific training.

## 6. Conclusion

This paper uses the multisensor information fusion technology method to realize the digital monitoring and intelligent decision-making of the fencing special ability training system to a certain extent, realize the quantification of the action and load of the special ability training, and realize the evaluation of the special ability training level and the decision of the load level. Additionally, various aspects are described, which are involved in the tracking of the load level trajectory, such as training load level diagnosis model and target decision model, identifying the training parameters that cause the training state to deviate from the normal load trajectory operating range, and instructing the athletes to adjust the training parameter changes accordingly. In the process of realizing decision-level data fusion, fuzzy rules under multiple conditions are designed, and the information of training parameters and training load is integrated by fuzzy inference, and the fusion result is used as the navigation instruction information for athletes to adjust training load. In the training process, the load level calculation and tracking are realized, and the ability level marked by the training load level is judged according to the fusion result, and the training target content is determined.

## Figures and Tables

**Figure 1:** Function of training target decision-making system.

**Figure 2:** The structure of the training target decision-making system.

**Figure 3:** Load level diagnosis and monitoring process.

**Figure 4:** Linguistic variable membership functions.

**Figure 5:** The load level relationship between the pedaling amplitude and the pedaling frequency.

**Figure 6:** Fuzzy set universe mapping.

**Figure 7:** Membership function of load class deviation.

**Figure 8:** Bias defuzzification.

**Figure 9:** Fuzzy monitoring of training load level and training parameters.

**Table 1:** Fuzzy rules for load changes.

Degree of load change	Heavy	Medium	Little
Speed control	Reduce	Keep	Increase
Force control	Reduce	Keep	Increase

**Table 2:** Fuzzy relationship between load level and training parameters.

Training requirements	Training parameters		
Load class	Pedal range	Pedaling frequency	Pedaling power
1	Low	Low	Low
2	Low	Middle	Low
	Middle	Low	Middle

3	Low	High	Low
	Middle	Middle	Middle
	High	Low	High

4	Middle	High	Middle
	High	Middle	High

5	High	High	High

**Table 3:** Control rule.

*e*	NB	NS	O	PS	PB
*u*	PB	PS	O	NS	NB

**Table 4:** Fuzzy variable (*e*, *u*) assignment table.

	−3	−2	−1	0	1	2	3
PB	0	0	0	0	0	0.4	0.8
PS	0	0	0	0	0.9	0.4	0
O	0	0.5	0.9	0.5	0.5	0.6	0
NS	0	0.4	1	0.6	0.4	0	0
NB	1	0.4	0.5	0	0	0	0

**Table 5:** Fusion results of fuzzy rules of types A and B.

Load level	Type A fuzzy rule fusion	Type B fuzzy rule fusion
1	*μ*_*A*1_(*z*)=*μ*_*A*1_(*w*_0_)∧*μ*_*A*1_(*f*_0_)=0	*μ*_*B*1_(*z*)=*μ*_*B*1_(*w*_0_)∧*μ*_*B*1_(*f*_0_)=0
2	$\begin{array}{c} \mu_{A2}\left(z\right)=\mu_{A1}\left(w_{0}\right)\wedge \mu_{A2}\left(f_{0}\right)=0.5\\ \mu_{A3}\left(z\right)=\mu_{A1}\left(w_{0}\right)\wedge \mu_{A3}\left(f_{0}\right)=0 \end{array}$	$\begin{array}{c} \mu_{B2}\left(z\right)=\mu_{B1}\left(w_{0}\right)\wedge \mu_{B2}\left(f_{0}\right)=0.5\\ \mu_{B3}\left(z\right)=\mu_{B1}\left(w_{0}\right)\wedge \mu_{B3}\left(f_{0}\right)=0 \end{array}$
3	$\begin{array}{c} \mu_{A4}\left(z\right)=\mu_{A2}\left(w_{0}\right)\wedge \mu_{A1}\left(f_{0}\right)=0\\ \mu_{A5}\left(z\right)=\mu_{A2}\left(w_{0}\right)\wedge \mu_{A2}\left(f_{0}\right)=0.5\\ \mu_{A6}\left(z\right)=\mu_{A2}\left(w_{0}\right)\wedge \mu_{A3}\left(f_{0}\right)=0 \end{array}$	$\begin{array}{c} \mu_{B4}\left(z\right)=\mu_{B2}\left(w_{0}\right)\wedge \mu_{B1}\left(f_{0}\right)=0\\ \mu_{B5}\left(z\right)=\mu_{B2}\left(w_{0}\right)\wedge \mu_{B2}\left(f_{0}\right)=1\\ \mu_{B6}\left(z\right)=\mu_{B2}\left(w_{0}\right)\wedge \mu_{B3}\left(f_{0}\right)=0 \end{array}$
4	$\begin{array}{c} \mu_{A7}\left(z\right)=\mu_{A3}\left(w_{0}\right)\wedge \mu_{A1}\left(f_{0}\right)=0\\ \mu_{A8}\left(z\right)=\mu_{A3}\left(w_{0}\right)\wedge \mu_{A2}\left(f_{0}\right)=0 \end{array}$	$\begin{array}{c} \mu_{B7}\left(z\right)=\mu_{B3}\left(w_{0}\right)\wedge \mu_{B1}\left(f_{0}\right)=0\\ \mu_{B8}\left(z\right)=\mu_{B3}\left(w_{0}\right)\wedge \mu_{B2}\left(f_{0}\right)=0 \end{array}$
5	*μ*_*A*9_(*z*)=*μ*_*A*3_(*w*_0_)∧*μ*_*A*3_(*f*_0_)=0	*μ*_*B*9_(*z*)=*μ*_*B*3_(*w*_0_)∧*μ*_*B*3_(*f*_0_)=0

## Data Availability

The datasets used and analyzed during the current study are available from the corresponding author upon reasonable request.
